# Modeling the Transmission Dynamics of Hepatitis A with Combined Vaccination and Sanitation Mitigation

**DOI:** 10.1155/2023/1203049

**Published:** 2023-02-13

**Authors:** Stephen Edward Mwaijande, Godfrey Edward Mpogolo

**Affiliations:** ^1^Department of Mathematics and Statistics, University of Dodoma, 338, Dodoma, Tanzania; ^2^Department of Management Studies, Tanzania Institute of Accountancy, 9522, Dar es Salaam, Tanzania

## Abstract

A mathematical model for the Hepatitis A Virus (HAV) epidemiology with dual transmission mechanisms is developed and presented. The model considers vaccination and sanitation as mitigation strategies. The effective reproductive number was derived and employed to study the stability of the model. Using Routh's stability criteria, the local stability of a disease-free equilibrium was determined, whereas the global stability of the endemic equilibrium was attained through a suitable Lyapunov function. Furthermore, bifurcation analysis is carried out using the centre manifold theory to ascertain its nature and implication for disease control. It was revealed that the model exhibits a forward bifurcation indicating the possibility of disease eradication when the effective reproduction number is kept below unity. Numerical results indicate that infection rates decrease quantitatively when at least one control measure is effectively implemented. It was deduced that combining vaccination and sanitation yields even fewer cases, making it the best alternative for eliminating Hepatitis A (HA) infection from the community. A sensitivity analysis was conducted to ascertain the parameters of the strong influence that could significantly affect the system. It was revealed that constant recruitment and vaccination coverage were the most critical parameters affecting the system. In addition, the study found that direct transmission plays an essential role in the occurrence of HA infection. In contrast, indirect transmission contributes marginally but significantly to the prevalence of HA infection.

## 1. Introduction

The hepatitis A virus (HAV) is the leading cause of acute liver infection known as viral hepatitis A. It is one of the earliest diseases that humans have ever encountered. Only a tiny percentage of people with this disease develops fulminant hepatitis and die. However, HAV is a significant contributor to morbidity and socioeconomic losses in many parts of the world. Hepatitis type A, infectious hepatitis, epidemic hepatitis, epidemic jaundice, and catarrhal jaundice were all previous names for the disease [1].

According to WHO estimates, 7134 people worldwide died from hepatitis A in 2016 (making up 0.5% of deaths from viral hepatitis) [1]. The overall case fatality rate is 0.3%, whereas the rate for humans aged 50 and older is 1.8%. Those with underlying chronic liver disease have a higher mortality risk [2]. Hepatitis A is a viral infection, so medications are ineffective against the disease. Antiviral agents and corticosteroids do not affect acute disease management. There is a trusted and safe vaccine available. Appropriate vaccine dosages and schedules throughout the first two years of life are needed to overcome the decreased immune response reported in infants who have passively acquired maternal anti-HAV.

The virus can be spread between humans via the fecal-oral pathway, by consuming contaminated foods or drinks, or by intravenous drug administration [3, 4]. Transmission is also possible with exposure to blood or blood products containing HAV but not saliva or urine. HA infection might also be transmitted through oral-anal sexual contact and blood transfusions. In particular, youngsters and asymptomatic and nonjaundiced HAV-infected persons are a significant source of HAV transmission [5]. Travel is another prominent source of infection in high-endemicity locations, where direct and indirect transmission may occur [6]. The typical incubation period (moment between exposure and onset of symptoms) is 28 days (ranging from 15 to 50 days), with infectivity peaking two weeks before the beginning of jaundice and dropping a week afterward [7].

Fever, anorexia, nausea, vomiting, diarrhea, myalgia, and malaise are among the warning symptoms of hepatitis A. Jaundice, dark-colored urine, or light-colored feces may be present at the onset of clinical symptoms or develop a few days later [8]. A sufficient supply of pure drinking water, proper sewage disposal within communities, and personal hygiene routines, like frequent hand washing, prevent the spread of HA infection [9]. A couple of decades ago, viral transmission decreased substantially in most developed nations due to improved living situations, sanitation, and environmental factors. These changes occurred without a specific vaccination strategy, highlighting the critical need for environmental and personal hygiene and sanitation.

Various mathematical models have been utilized to explore the dynamics of HAV transmission and the viability of mitigation strategies for HA outbreaks.

Guimaraens and Codeço [10] established a susceptible-infectious-recovery (SIR) mathematical model to examine the impact of varying infection exposures on the epidemiological dynamics of hepatitis A. Their research has found that uneven access to sanitary facilities is a hallmark of Brazilian communities. This heterogeneity leads to distinct patterns of hepatitis A endemicity: places with low infection rates have a greater likelihood of outbreaks, whereas locations with high infection rates have a greater incidence and a reduced risk of epidemics. Also, a mathematical model that considers susceptible, latent, infectious, and recovered-immune (S-L-I-R) was designed to underscore the urgency of considering herd protection triggered by early childhood HA immunization [11]. The model supported the recommendations of the Immunization Practices Advisory Committee for universal HA vaccination of one-year-olds [12].

On the other hand, another work was by [13], where the basic mathematical model for the temporal dynamics of HAV in Italy regions with a moderate endemicity was established. This study presented three transmission mechanisms: direct transmission between susceptible and infectious persons, indirect transmission through the consumption of locally infected food, and migration to highly endemic regions. Consideration was given to a periodicity in indirect transmission, as evidenced by statistics on fishing and the eating of shellfish. Vaccination of infants and adults, similar to the program already in effect in Puglia, was also included.

Likewise, [14] developed an individual-based model with a dynamic network of linkages that were parameterized using sociodemographic and epidemiologic data and accounted for millions of people. The research concluded that the low vaccination rate in Italy is adequate to prevent the emergence of hepatitis A. Nevertheless, eradication is impossible because of the continuous influx of new cases from highly endemic locations outside the country.

Moreover, [15] built and calibrated a compartmental dynamic transmission model stratified by age and context in rural and urban Thailand, utilizing demographic, environmental, and epidemiological data. This model was used to project several epidemiological measures. Their research suggests a novel method for assessing HAV epidemiological patterns and future projections considering the interaction between water, urbanization, and endemicity. This method provides insights into the developing HAV epidemiology and might be used to examine the public health impact of vaccination and other therapies in various settings.

Recently, scholars such as in [16, 17] have also studied the dynamics and the effects of a vaccination strategy in containing HA infection. In particular, [16] developed a mathematical model of HAV transmission to assess trends of regional spread and the effect of vaccination on the extent and timing of the HAV outbreak in Michigan. Specifically, they evaluated the proportion of cases prevented by the vaccination program in Southeast Michigan and the remainder of the state. However, [17] established a linear age-structured SEIAR (susceptible-exposed-symptomatic-asymptomatic-recovered) compartmental model to examine the dynamics and effects of various vaccination approaches on HAV evolution.

This study was inspired by the work of [13]. Nevertheless, their research did not account for the role of sanitation strategy in the control of HAV. Therefore, the central purpose of this work was to develop a dynamic deterministic epidemiological model that considers both direct and indirect mechanisms of HAV transmission in the presence of vaccination and sanitation control efforts.

The paper has the following structure. The second section is devoted to the model formulation. In contrast, the third section analyzes the model, Section 4 then addresses the numerical simulation, Section 5 is dedicated to sensitivity analysis, and Section 6 concludes the paper with final remarks.

## 2. Model Formulation

This section develops a deterministic epidemiological model that tracks the HAV transmission process. The epidemiology of this disease ensures an incubation time. Therefore, the work of [13] is expanded by including an additional compartment for the exposed population. Furthermore, the notion of a dynamic system is incorporated into this model. Since a static population is implausible, the death rate should be distinct from the birth rate to allow for a dynamic system. As in [13], the current model will incorporate the following transmission routes: human-to-human transmission (direct path) and environment-to-human transmission (indirect path). Besides that, unlike [13], our model incorporates multiple control initiatives: vaccination and sanitation.

The total population is subdivided into six mutually exclusive epidemiological classes: susceptible *S*(*t*), vaccinated *V*(*t*), latent *L*(*t*), infectious *I*(*t*), and recovered *R*(*t*). We extend the SIR model by introducing the following classes: *L*(*t*), *V*(*t*), and *P*(*t*), where *P*(*t*) represents the pool of HA pathogens in food or water.

It is credible to hypothesize that susceptible humans join the community at a constant rate *Λ*. At the time-dependent rates *λ*_1_(*t*) and *λ*_2_(*t*), susceptible humans may become infected after direct contact with infectious humans or after ingesting pathogens from contaminated food or water, respectively. Specifically, *λ*_1_(*t*) denotes direct transmission among humans, while *λ*_2_(*t*) denotes indirect transmission, both modeled by the bilinear incidence rate. The overall force of infection is shown by the symbol *λ*(*t*) and is defined by

(1) $$\begin{array}{c} \lambda \left(t\right)=\lambda_{1}\left(t\right)+\lambda_{2}\left(t\right), \end{array}$$

where

(2) $$\begin{array}{c} \begin{array}{c} \lambda_{1}\left(t\right)=\beta_{1}I\left(t\right),\\ \lambda_{2}\left(t\right)=\beta_{2}P\left(t\right). \end{array} \end{array}$$

Further, *β*_1_ stands for the transmission rate for infectious humans, while *β*_2_ stands for the ingestion rate of HA pathogens by humans. Humans in the exposed stage move to the infectious stage at the rate *α*. Since no treatment is available for this disease, we assume that once infected, humans may recover naturally at the rate *γ*. Any individual in the population is considered to have a possibility of undergoing natural mortality whose rate is represented by *μ*. Also, HAV infection is known to confer permanent immunity upon recovery. Thus, recovering humans are not expected to rejoin the susceptible class. According to the disease epidemiology, it is known that infected humans may shed the virus to the surroundings, which could spoil food or water that humans could later consume. Thus, we assume that infectious humans may shed the virus to the surroundings at the rate *δ*. HA viruses' per capita growth rate is represented by *ϕ*, whereas viruses die naturally at the rate *μ*_*p*_ or by sanitation efforts at the rate *η*. The growth rate of viruses *ϕ* is expected not to surpass its death rate *μ*_*p*_. The variables and parameters that the model will utilize have been outlined in detail in Tables 1 and 2, respectively.  Figure 1 depicts the flowchart for the dynamics of HAV.

Integrating Figure 1, model assumptions, and the model description yield the system differential equations:

(3) $$\begin{array}{c} \begin{array}{c} \frac{dS}{dt}=\left(1-\rho \right)\Lambda -\left(\mu +\theta +\lambda \right)S,\\ \frac{dV}{dt}=\rho \Lambda +\theta S-\mu V,\\ \frac{dL}{dt}=\lambda S-\left(\mu +\alpha \right)L,\\ \frac{dI}{dt}=\alpha L-\left(\mu +\gamma +\delta \right)I,\\ \frac{dR}{dt}=\gamma I-\mu R,\\ \frac{dP}{dt}=\delta I-\left(\mu_{p}+\eta -\phi \right)P. \end{array} \end{array}$$

The model system's initial conditions can be considered as *S*(0) > 0, *L*(0) > 0, *I*(0) > 0, *V*(0) > 0, *R*(0) > 0, *P*(0) > 0.

## 3. Analysis of the Model

### 3.1. Boundedness of Solutions

The model system (3) can be split into two parts which include the human population *T*_*H*_ and the density of viruses in the surroundings (food/water) *T*_*P*_ such that *T*_*H*_ = {(*S*(*t*), *L*(*t*), *I*(*t*), *V*(*t*), *R*(*t*)) ∈ ℝ_+_^5^ : *S*(*t*) + *V*(*t*) + *L*(*t*) + *I*(*t*) + *R*(*t*) = *N*(*t*)} and *T*_*P*_ = {*P*(*t*) ∈ ℝ_+_^1^}, respectively. From the model system (3), the differential inequality of the susceptible population is given by

(4) $$\begin{array}{c} \frac{dS}{dt}+\left(\mu +\theta +\lambda \right)S=\left(1-\rho \right)\Lambda . \end{array}$$

Solving equation (4), one gets

(5) $$\begin{array}{c} S\left(t\right)\leq \frac{\left(1-\rho \right)\Lambda }{\mu +\theta +\lambda }+e^{-\left(\mu +\theta +\lambda \right)t}\int_{0}^{t}\phi V\left(x\right)e^{-\left(\mu +\theta +\lambda \right)x}dx. \end{array}$$

By adopting Birkhoff and Rota's theorem of differential inequality [21], we have

(6) $$\begin{array}{c} \underset{t⟶\infty }{\lim}\sup S\left(t\right)\leq \frac{\left(1-\rho \right)\Lambda }{\mu +\theta +\lambda }. \end{array}$$

We observe that the population in total is represented as *N* = *S* + *V* + *L* + *I* + *R*. Thus, one may use system (3) to establish the formula:

(7) $$\begin{array}{c} \frac{dN}{dt}=\Lambda -\mu N. \end{array}$$

The solution to equation (7) at *N*(0) = *N*^0^ gives

(8) $$\begin{array}{c} N\left(t\right)=\frac{\Lambda }{\mu }-\left(\frac{\Lambda }{\mu }-N^{0}\right)e^{-\mu t}. \end{array}$$

Therefore,

(9) $$\begin{array}{c} \underset{t⟶\infty }{\lim}\sup N\left(t\right)\leq \frac{\Lambda }{\mu }. \end{array}$$

So long as *N* represents the total population, then every state variable has a value below or equivalent to *Λ*/*μ*. Also, applying the assumption that the HA pathogen's growth rate is lesser than its fatality rate (i.e., *ϕ* < *μ*_*p*_), the equation for *P* from the system (3) becomes

(10) $$\begin{array}{c} \frac{dP}{dt}+\left(\mu_{p}+\eta -\phi \right)P=\delta I\leq \frac{\delta \Lambda }{\mu }. \end{array}$$

On solving equation (10), one obtains

(11) $$\begin{array}{c} \underset{t⟶\infty }{\lim}\sup P\left(t\right)\leq \frac{\delta \Lambda }{\mu \left(\mu_{p}+\eta -\phi \right)}. \end{array}$$

Consequently, the system's region of biological relevance (3) is

(12) $$\begin{array}{c} T=\left[S,V,L,I,R,P\geq 0:S+V+L+I+R\leq \frac{\Lambda }{\mu },P\leq \frac{\delta \Lambda }{\mu \left(\mu_{p}+\eta -\phi \right)}\right]. \end{array}$$

The region *T* is positively invariant under the flow induced by the system (3). Therefore, the system (3) is biologically meaningful, and it is feasible to analyze the model in the domain *T*.

### 3.2. Existence of Equilibrium Solutions

In the current section, we derive the conditions for the existence of the equilibria. This will be achieved by setting the right-hand side of the system (3) to zero and solving the resulting system:

(13) $$\begin{array}{c} \begin{array}{c} 0=\left(1-\rho \right)\Lambda -\left(\lambda^{*}+\mu +\theta \right)S^{*},\\ 0=\rho \Lambda +\theta S^{*}-\mu V^{*},\\ 0=\lambda^{*}S^{*}-\left(\mu +\alpha \right)L^{*},\\ 0=\alpha L^{*}-\left(\mu +\gamma +\delta \right)I^{*},\\ 0=\gamma I^{*}-\mu R^{*},\\ 0=\delta I^{*}-\left(\mu_{p}+\eta -\phi \right)P^{*}, \end{array} \end{array}$$

where

(14) $$\begin{array}{c} \begin{array}{c} \lambda^{*}=\beta_{1}I^{*}+\beta_{2}P^{*}. \end{array} \end{array}$$

Solving the system (13) in terms of *L*^∗^, we get

(15) $$\begin{array}{c} \begin{array}{c} S^{*}=\frac{\left(1-\rho \right)\Lambda -\left(\mu +\alpha \right)L^{*}}{\mu +\theta },\\ V^{*}=\frac{\left(1-\rho \right)\Lambda \theta -\left(\mu +\alpha \right)L^{*}}{\mu +\theta },\\ I^{*}=\frac{\alpha L^{*}}{\left(\mu +\gamma +\delta \right)},\\ R^{*}=\frac{\alpha \gamma L^{*}}{\mu \left(\mu +\gamma +\delta \right)},\\ P^{*}=\frac{\alpha \delta L^{*}}{\left(\mu_{p}+\eta -\phi \right)\left(\mu +\gamma +\delta \right)}. \end{array} \end{array}$$

To obtain *L*^∗^, one can express

(16) $$\begin{array}{c} \lambda^{*}=Q_{4}L^{*}, \end{array}$$

where

(17) $$\begin{array}{c} Q_{4}=\frac{\alpha \left(\beta_{1}\left(\mu_{p}+\eta -\phi \right)+\beta_{2}\delta \right)}{\left(\mu_{p}+\eta -\phi \right)\left(\mu +\gamma +\delta \right)}. \end{array}$$

Put *λ*^∗^, *S*^∗^, and *L*^∗^ to the third equation of the system (13) to get

(18) $$\begin{array}{c} Q_{4}L^{*}\left(\frac{\left(1-\rho \right)\Lambda -\left(\mu +\alpha \right)L^{*}}{\mu +\theta }\right)=\left(\mu +\alpha \right)L^{*}, \end{array}$$

(19) $$\begin{array}{c} Q_{4}\left(\left(1-\rho \right)\Lambda -\left(\mu +\alpha \right)L^{*}\right)L^{*}-\left(\mu +\theta \right)\left(\mu +\alpha \right)L^{*}=0, \end{array}$$

(20) $$\begin{array}{c} Q_{4}\left(\mu +\alpha \right){L^{*}}^{2}+\left(\left(\mu +\theta \right)\left(\mu +\alpha \right)-Q_{4}\left(1-\rho \right)\Lambda \right)L^{*}=0, \end{array}$$

(21) $$\begin{array}{c} A{L^{*}}^{2}+BL^{*}+C=0, \end{array}$$

where

(22) $$\begin{array}{c} \begin{array}{c} A=Q_{4}\left(\mu +\alpha \right)=\frac{\alpha \left(\mu +\alpha \right)\left(\beta_{1}\left(\mu_{p}+\eta -\phi \right)+\beta_{2}\delta \right)}{\left(\mu_{p}+\eta -\phi \right)\left(\mu +\gamma +\delta \right)},\\ B=\left(\mu +\theta \right)\left(\mu +\alpha \right)\left(1-R_{e}\right),\\ C=0. \end{array} \end{array}$$

Equation (20) has two solutions:

(23) $$\begin{array}{c} \begin{array}{c} L^{*}=0,\\ L^{*}=-\frac{B}{A}=\frac{\left(\mu +\theta \right)}{Q_{4}}\left(R_{e}-1\right)=\frac{\left(\mu +\theta \right)\left(\mu_{p}+\eta -\phi \right)\left(\mu +\gamma +\delta \right)}{\alpha \left(\beta_{1}\left(\mu_{p}+\eta -\phi \right)+\beta_{2}\delta \right)}\left(R_{e}-1\right), \end{array} \end{array}$$

where

(24) $$\begin{array}{c} R_{e}=\frac{Q_{4}\left(1-\rho \right)\Lambda }{\left(\mu +\theta \right)\left(\mu +\alpha \right)}=\frac{\alpha \beta_{1}\left(1-\rho \right)\Lambda }{\left(\mu +\alpha \right)\left(\mu +\gamma +\delta \right)\left(\mu +\theta \right)}+\frac{\alpha \delta \beta_{2}\left(1-\rho \right)\Lambda }{\left(\mu +\alpha \right)\left(\mu +\gamma +\delta \right)\left(\mu_{p}+\eta -\phi \right)\left(\mu +\theta \right)}. \end{array}$$

It should be observed that the presence of a disease-free state coincides with *L*^∗^ = 0, whereas

(25) $$\begin{array}{c} \begin{array}{c} L^{*}=\frac{\left(\mu +\theta \right)\left(\mu_{p}+\eta -\phi \right)\left(\mu +\gamma +\delta \right)}{\alpha \left(\beta_{1}\left(\mu_{p}+\eta -\phi \right)+\beta_{2}\delta \right)}\left(R_{e}-1\right) \end{array} \end{array}$$

coincides with the persistence of the endemic equilibrium point; in fact, *L*^∗^ > 0, whenever *R*_*e*_ > 1.

#### 3.2.1. Disease-Free Equilibrium (DFE) Point

In the absence of infection, a disease-free equilibrium is achieved. Therefore, *L*_0_^∗^ = 0 represents the state of the DFE. Putting *L*_0_^∗^ = 0 into equation (15), one obtains the DFE:

(26) $$\begin{array}{c} E_{0}=\left(S_{0}^{*},V_{0}^{*},L_{0}^{*},I_{0}^{*},R_{0}^{*},P_{0}^{*}\right)=\left(\frac{\left(1-\rho \right)\Lambda }{\mu +\theta },\frac{\left(1-\rho \right)\Lambda \theta }{\mu +\theta },0,0,0,0\right). \end{array}$$

#### 3.2.2. Endemic Equilibrium (EE) Point

The endemic equilibrium point is the nonzero equilibrium solution of the model system (3). It is achieved when *S*^∗^, *V*^∗^, *L*^∗^, *I*^∗^, *R*^∗^, *P*^∗^ > 0. In this scenario, the nontrivial value of *L*^∗^ from equation (25) is substituted into equation (15) to obtain an EE point

(27) $$\begin{array}{c} E_{1}=\left(S^{*},V^{*},L^{*},I^{*},R^{*},P^{*}\right), \end{array}$$

where

(28) $$\begin{array}{c} \begin{array}{c} S^{*}=\frac{\left(1-\rho \right)\Lambda Q_{4}-\left(\mu +\theta \right)\left(\mu +\alpha \right)\left(R_{e}-1\right)}{\left(\mu +\theta \right)Q_{4}},\\ V^{*}=\frac{\left(1-\rho \right)\Lambda \theta Q_{4}-\left(\mu +\theta \right)\left(\mu +\alpha \right)\left(R_{e}-1\right)}{\left(\mu +\theta \right)Q_{4}},\\ L^{*}=\frac{\left(\mu +\theta \right)}{Q_{4}}\left(R_{e}-1\right),\\ I^{*}=\frac{\alpha \left(\mu +\theta \right)\left(R_{e}-1\right)}{\left(\mu +\gamma +\delta \right)Q_{4}},\\ R^{*}=\frac{\alpha \gamma \left(\mu +\theta \right)\left(R_{e}-1\right)}{\mu \left(\mu +\gamma +\delta \right)Q_{4}},\\ P^{*}=\frac{\alpha \delta \left(\mu +\theta \right)\left(R_{e}-1\right)}{\left(\mu_{p}+\eta -\phi \right)\left(\mu +\gamma +\delta \right)Q_{4}}. \end{array} \end{array}$$

Clearly, the endemic equilibrium exists provided *R*_*e*_ > 1.

### 3.3. The Effective Reproduction Number and Stability Analysis of Equilibria

The average number of secondary infections someone generates throughout their whole infectious lifetime is reflected by the effective reproduction number, *R*_*e*_ [22]. It establishes the threshold at which disease can be predicted to spread or vanish in the community, and it also can aid in evaluating the feasibility of control strategies. In addition, through *R*_*e*_, stability analysis of equilibrium is possible. If *R*_*e*_ < 1, each infectious individual will only generate a single secondary infection, leading to the extinction of the disease. If *R*_*e*_ > 1, each contagious person will spread the disease across the community by causing several secondary infections. A high value of *R*_*e*_ could portend the potential for a significant disease epidemic.

Using a similar technique to the one employed in the work by [23], we establish the effective reproduction number, *R*_*e*_. The matrix's dominant (maximum) eigenvalue (spectral radius) is used to calculate the effective reproduction number. The effective reproduction number is determined through the largest (dominant) eigenvalue (spectral radius) of the matrix

(29) $$\begin{array}{c} \text{F}{\text{V}}^{-1}=\left[\frac{\partial F_{i}\left(E_{0}\right)}{\partial x_{j}}\right]{\left[\frac{\partial V_{i}\left(E_{0}\right)}{\partial x_{j}}\right]}^{-1}. \end{array}$$

The rate for which new cases arise in compartment *i* is determined by *F*_*i*_, whereas the rate at which infections propagate from one compartment to the next is determined by *V*_*i*_, whereas *E*_0_ stands for DFE. Considering the equations for infected compartments, *L*, *I*, *C*, and *B* from system (3) give

(30) $$\begin{array}{c} \begin{array}{c} \frac{dL}{dt}=\lambda S-\left(\mu +\alpha \right)L,\\ \frac{dI}{dt}=\alpha L-\left(\mu +\gamma +\delta \right)I,\\ \frac{dP}{dt}=\delta I-\left(\mu_{p}+\eta -\phi \right)P, \end{array} \end{array}$$

where *λ* = *β*_1_*I* + *β*_2_*P*.

Let

(31) $$\begin{array}{c} \begin{array}{c} A_{11}=\mu +\alpha ,\\ A_{12}=\beta_{1}S^{0},\\ A_{13}=\beta_{2}S^{0},\\ A_{21}=\alpha ,\\ A_{22}=\mu +\gamma +\delta ,\\ A_{32}=\delta ,\\ A_{33}=\mu_{p}+\eta -\phi . \end{array} \end{array}$$

From the system (30), we obtain

(32) $$\begin{array}{c} F_{i}=\left[\begin{array}{c} \beta_{1}\text{SI}+\beta_{2}\text{SP}\\ 0\\ 0 \end{array}\right],\\ V_{i}=\left[\begin{array}{c} A_{11}L\\ A_{22}I-A_{21}L\\ A_{33}P-A_{32}I \end{array}\right]. \end{array}$$

Partially differentiating *F*_*i*_ and *V*_*i*_ with respect to *L*, *I*, and *P* and evaluating at DFE result in

(33) $$\begin{array}{c} F=\left[\begin{array}{ccc} 0 & A_{12} & A_{13}\\ 0 & 0 & 0\\ 0 & 0 & 0 \end{array}\right], \end{array}$$

(34) $$\begin{array}{c} V=\left[\begin{array}{ccc} A_{11} & 0 & 0\\ -A_{21} & A_{22} & 0\\ 0 & -A_{32} & A_{33} \end{array}\right], \end{array}$$

(35) $$\begin{array}{c} V^{-1}=\left[\begin{array}{ccc} {A_{11}}^{-1} & 0 & 0\\ \frac{A_{21}}{A_{11}A_{22}} & {A_{22}}^{-1} & 0\\ \frac{A_{21}A_{32}}{A_{11}A_{22}A_{33}} & \frac{A_{32}}{A_{22}A_{33}} & {A_{33}}^{-1} \end{array}\right]. \end{array}$$

The effective reproduction number is now given by

(36) $$\begin{array}{c} R_{e}=\rho \left(FV^{-1}\right)=\frac{A_{21}A_{12}}{A_{22}A_{11}}+\frac{A_{32}A_{21}A_{13}}{A_{33}A_{22}A_{11}},\\ R_{e}=R_{01}+R_{02}, \end{array}$$

where

(37) $$\begin{array}{c} \begin{array}{c} R_{01}=\frac{A_{21}A_{12}}{A_{22}A_{11}},\\ R_{02}=\frac{A_{32}A_{21}A_{13}}{A_{33}A_{22}A_{11}}. \end{array} \end{array}$$

Substituting values of *A*_*ij*_, ∀*i*, *j* = 1, 2, 3, from equation (31), we get

(38) $$\begin{array}{c} R_{e}=\frac{\alpha \beta_{1}\left(1-\rho \right)\Lambda }{\left(\mu +\alpha \right)\left(\mu +\gamma +\delta \right)\left(\mu +\theta \right)}+\frac{\alpha \delta \beta_{2}\left(1-\rho \right)\Lambda }{\left(\mu +\alpha \right)\left(\mu +\gamma +\delta \right)\left(\mu_{p}+\eta -\phi \right)\left(\mu +\theta \right)}. \end{array}$$

Moreover, *R*_01_ and *R*_02_ represent the contributions via direct and indirect transmissions, respectively.

### 3.4. Local Stability of Disease-Free Equilibrium

Here, we establish the local stability of disease-free equilibrium (26) using Routh's stability criterion.

**Theorem 1 .**

The DFE of the model system (3) is locally asymptotically stable if *R*_*e*_ < 1 and unstable if *R*_*e*_ > 1.

**Proof**

The partial differentiation of system (3) with respect to (*S*, *V*, *L*, *I*, *R*, *P*) at the disease-free equilibrium gives the Jacobian matrix *J* as

(39) $$\begin{array}{c} J\left(E_{0}\right)=\left[\begin{array}{cccccc} -\left(\mu +\theta \right) & 0 & 0 & -\beta_{1}S_{0} & 0 & -\beta_{2}S_{0}\\ \theta & -\mu & 0 & 0 & 0 & 0\\ 0 & 0 & -\mu -\alpha & \beta_{1}S_{0} & 0 & \beta_{2}S_{0}\\ 0 & 0 & \alpha & -\mu -\gamma -\delta & 0 & 0\\ 0 & 0 & 0 & \gamma & -\mu & 0\\ 0 & 0 & 0 & \delta & 0 & -\mu_{p}-\eta +\phi \end{array}\right]. \end{array}$$

The matrix (39) has three trivial negative eigenvalues *λ* = −*μ*, *λ* = −(*μ* + *θ*), and *λ* = −*μ*.

To find the rest eigenvalues, we consider a submatrix *J*_1_ as follows:

(40) $$\begin{array}{c} J_{1}\left(E_{0}\right)=\left[\begin{array}{ccc} -\mu -\alpha & \beta_{1}S_{0}^{*} & \beta_{2}S_{0}^{*}\\ \alpha & -\mu -\gamma -\delta & 0\\ 0 & \delta & -\mu_{p}-\eta +\phi \end{array}\right]=\left[\begin{array}{ccc} -A_{11} & A_{12} & A_{13}\\ A_{21} & -A_{22} & 0\\ 0 & A_{32} & -A_{33} \end{array}\right], \end{array}$$

where *A*_11_, *A*_12_, *A*_13_, *A*_21_, *A*_22_, *A*_32_, *A*_33_ are defined from equation (31).

We derive the characteristic polynomial using matrix (40) and get the following:

(41) $$\begin{array}{c} c_{0}\lambda^{3}+c_{1}\lambda^{2}+c_{2}\lambda +c_{3}=0, \end{array}$$

where

(42) $$\begin{array}{c} \begin{array}{c} c_{0}=1,\\ c_{1}=A_{33}+A_{22}+A_{11},\\ c_{2}=A_{33}A_{22}+A_{33}A_{11}+A_{22}A_{11}\left(1-R_{01}\right),\\ c_{3}=A_{33}A_{22}A_{11}\left(1-R_{e}\right),\\ R_{e}=R_{01}+R_{02},\\ R_{01}=\frac{A_{21}A_{12}}{A_{22}A_{11}},\\ R_{02}=\frac{A_{32}A_{21}A_{13}}{A_{33}A_{22}A_{11}}. \end{array} \end{array}$$

Since we have a polynomial of degree 3, then Routh's stability criterion states that all roots possess negative real parts if and only if

1. all the *c*_*i*_ (*i* = 0, 1, 2, 3) are positive,
2. *c*_1_*c*_2_ > *c*_0_*c*_3_.

It can be noted that *c*_0_ = 1 > 0, *c*_1_ > 0; moreover, *c*_2_, *c*_3_ > 0 provided *R*_01_, *R*_*e*_ < 1; therefore, all the *c*_*i*_ are positive. Consider

(43) $$\begin{array}{c} \begin{array}{c} c_{1}c_{2}=\left(A_{11}+A_{22}+A_{33}\right)\left(A_{11}A_{33}+A_{22}A_{33}+A_{11}A_{22}\left(1-R_{01}\right)\right),\\ c_{0}c_{3}=A_{11}A_{22}A_{33}\left(1-R_{e}\right). \end{array} \end{array}$$

Clearly, *c*_1_*c*_2_ > *c*_0_*c*_3_ only if *R*_01_ < *R*_*e*_ < 1. Hence, the DFE is locally asymptotically stable since the roots of equation (41) have negative real parts whenever *R*_*e*_ < 1.

An application of Routh-Hurwitz criteria gives *R*_*e*_(*λ*) < 0 if and only if

(44) $$\begin{array}{c} c_{3}>0, \end{array}$$

(45) $$\begin{array}{c} c_{2}c_{3}>c_{0}c_{3}. \end{array}$$

### 3.5. Global Stability of Disease-Free Equilibrium Point

Below is the finding concerning the global stability of the disease-free equilibrium; a comparison approach is employed to reach this result.

**Theorem 2 .**

The disease-free equilibrium point is globally asymptotically stable if *R*_*e*_ < 1 and unstable otherwise.

**Proof**

Using the comparison theorem, we have

(46) $$\begin{array}{c} \left(\begin{array}{c} \frac{dL}{dt}\\ \frac{dI}{dt}\\ \frac{dP}{dt} \end{array}\right)=\left(F-V\right)\left(\begin{array}{c} L\\ I\\ P \end{array}\right)-\left(\begin{array}{ccc} 0 & \beta_{1}S_{0}^{*} & \beta_{2}S_{0}^{*}\\ 0 & 0 & 0\\ 0 & 0 & 0 \end{array}\right)\left(\begin{array}{c} L\\ I\\ P \end{array}\right), \end{array}$$

indicating that

(47) $$\begin{array}{c} \left(\begin{array}{c} \frac{dL}{dt}\\ \frac{dI}{dt}\\ \frac{dP}{dt} \end{array}\right)\leq \left(F-V\right)\left(\begin{array}{c} L\\ I\\ P \end{array}\right), \end{array}$$

where *F* and *V* are defined in (33) and (34).

It can be noted that the Jacobian matrix (*F* − *V*) is equivalent to the one in equation (40), which was proven in Theorem1 to contain all negative eigenvalues. Hence, (*S*, *V*, *L*, *I*, *R*, *P*)⟶(*S*^0^, *V*^0^, 0, 0, 0, 0) and *S*⟶*S*_0_ as *t*⟶∞. Therefore, *E*_0_ is globally asymptotically stable whenever *R*_*e*_ < 1.

### 3.6. Local Stability of Endemic Equilibrium

In the presence of infection, all the state variables for infected individuals, including the class for the HA virus, will be nonzero (this comes from the condition established in (25)). Thus, we express endemic equilibrium *E*_1_ in terms of *R*_*e*_ as follows: *E*_1_(*S*^∗^, *V*^∗^, *L*^∗^, *I*^∗^, *R*^∗^, *P*^∗^), where

(48) $$\begin{array}{c} \begin{array}{c} S^{*}=\frac{\left(1-\rho \right)\Lambda Q_{4}-\left(\mu +\theta \right)\left(\mu +\alpha \right)\left(R_{e}-1\right)}{\left(\mu +\theta \right)Q_{4}},\\ V^{*}=\frac{\left(1-\rho \right)\Lambda \theta Q_{4}-\left(\mu +\theta \right)\left(\mu +\alpha \right)\left(R_{e}-1\right)}{\left(\mu +\theta \right)Q_{4}},\\ L^{*}=\frac{\left(\mu +\theta \right)}{Q_{4}}\left(R_{e}-1\right),\\ I^{*}=\frac{\alpha \left(\mu +\theta \right)\left(R_{e}-1\right)}{\left(\mu +\gamma +\delta \right)Q_{4}},\\ R^{*}=\frac{\alpha \gamma \left(\mu +\theta \right)\left(R_{e}-1\right)}{\mu \left(\mu +\gamma +\delta \right)Q_{4}},\\ P^{*}=\frac{\alpha \delta \left(\mu +\theta \right)\left(R_{e}-1\right)}{\left(\mu_{p}+\eta -\phi \right)\left(\mu +\gamma +\delta \right)Q_{4}}. \end{array} \end{array}$$

We can establish the following result from equation (48).

**Theorem 3 .**

The endemic equilibrium for the model (3) is locally asymptotically stable on *T* if *R*_*e*_ > 1.

### 3.7. Global Stability of Endemic Equilibrium

In this section, the global stability of the endemic equilibrium point is carried out via a suitable choice of the Lyapunov function.

**Theorem 4 .**

The endemic equilibrium for the model (3) is globally asymptotically stable on *T* if *R*_*e*_ > 1.

**Proof**

Consider a Lyapunov function:

(49) $$\begin{array}{c} W=\overset{n}{\underset{i=1}{\sum }}k_{i}\left(x_{i}-x_{i}^{*}lnx\right), \end{array}$$

where *k*_*i*_ is a properly selected positive constant, *x*_*i*_ is the population of the *i*th compartment, and *x*_*i*_^∗^ is the equilibrium level. We define the Lyapunov function candidate *W* for model system (3) as

(50) $$\begin{array}{c} W=k_{1}\left(S-S^{*}lnS\right)+k_{2}\left(V-V^{*}lnV\right)+k_{3}\left(L-L^{*}lnL\right)+k_{4}\left(I-I^{*}lnI\right)+k_{5}\left(R-R^{*}lnR\right)+k_{6}\left(P-P^{*}lnP\right). \end{array}$$

The time derivative of the Lyapunov function *W* is given by

(51) $$\begin{array}{c} \frac{dW}{dt}=k_{1}\left(1-\frac{S^{*}}{S}\right)\frac{dS}{dt}+k_{2}\left(1-\frac{V^{*}}{V}\right)\frac{dV}{dt}+k_{3}\left(1-\frac{L^{*}}{L}\right)\frac{dL}{dt}+k_{4}\left(1-\frac{I^{*}}{I}\right)\frac{dI}{dt}+k_{5}\left(1-\frac{R^{*}}{R}\right)\frac{dR}{dt}+k_{6}\left(1-\frac{P^{*}}{P}\right)\frac{dP}{dt}. \end{array}$$

It can be noted that at the endemic equilibrium (see equation (13)), we have

(52) $$\begin{array}{c} \begin{array}{c} \left(1-\rho \right)\Lambda =\left(\lambda^{*}+\mu +\theta \right)S^{*},\rho \Lambda =\mu V^{*}-\theta S^{*},\mu +\alpha =\frac{\lambda^{*}S^{*}}{L^{*}},\\ \mu +\gamma +\delta =\frac{\alpha L^{*}}{I^{*}},\mu =\frac{\gamma I^{*}}{R^{*}},\mu_{p}+\eta -\phi =\frac{\delta I^{*}}{P^{*}}. \end{array} \end{array}$$

Substituting equation (52) into equation (51) and simplifying gives an equation:

(53) $$\begin{array}{c} \frac{dW}{dt}=-k_{2}\theta S\left(1-\frac{S^{*}}{S}\right)\left(1-\frac{V^{*}}{V}\right)-k_{1}\lambda S\left(1-\frac{S^{*}}{S}\right)\left(1-\frac{\lambda^{*}S^{*}}{\lambda S}\right)-k_{1}\left(\mu +\theta \right)S{\left(1-\frac{S^{*}}{S}\right)}^{2}-k_{2}\mu V{\left(1-\frac{V^{*}}{V}\right)}^{2}+k_{3}\lambda S\left(1-\frac{\lambda^{*}}{\lambda }\frac{S^{*}}{S}\frac{L}{L^{*}}\right)+k_{4}\alpha L\left(1-\frac{L^{*}}{L}\frac{I}{I^{*}}\right)+k_{5}\gamma I\left(1-\frac{I^{*}R}{IR^{*}}\right)+k_{6}\delta I\left(1-\frac{I^{*}P}{IP^{*}}\right), \end{array}$$

which can also be written as

(54) $$\begin{array}{c} \frac{dW}{dt}=-k_{2}\theta S\left(1-\frac{S^{*}}{S}\right)\left(1-\frac{V^{*}}{V}\right)-k_{1}\lambda S\left(1-\frac{S^{*}}{S}\right)\left(1-\frac{\lambda^{*}S^{*}}{\lambda S}\right)-k_{1}\left(\mu +\theta \right)S{\left(1-\frac{S^{*}}{S}\right)}^{2}-k_{2}\mu V{\left(1-\frac{V^{*}}{V}\right)}^{2}+F\left(S,V,L,I,R,P\right), \end{array}$$

where

(55) $$\begin{array}{c} F\left(S,V,L,I,R,P\right)=k_{3}\lambda S\left(1-\frac{\lambda^{*}}{\lambda }\frac{S^{*}}{S}\frac{L}{L^{*}}\right)+k_{4}\alpha L\left(1-\frac{L^{*}}{L}\frac{I}{I^{*}}\right)+k_{5}\gamma I\left(1-\frac{I^{*}R}{IR^{*}}\right)+k_{6}\delta I\left(1-\frac{I^{*}P}{IP^{*}}\right). \end{array}$$

Choose

(56) $$\begin{array}{c} \begin{array}{c} k_{1}=k_{3}=\frac{1}{\lambda S},\\ k_{2}=\frac{1}{\theta S},\\ k_{4}=\frac{1}{\alpha L},\\ k_{5}=\frac{1}{\delta I},\\ k_{6}=\frac{1}{\sigma I}, \end{array} \end{array}$$

then equation (54) becomes

(57) $$\begin{array}{c} \frac{dW}{dt}=-\frac{\left(\mu +\theta \right)}{\lambda }{\left(1-\frac{S^{*}}{S}\right)}^{2}-\frac{\mu V}{\theta S}{\left(1-\frac{V^{*}}{V}\right)}^{2}-\left(1-\frac{S^{*}}{S}\right)\left(2+\frac{V^{*}}{V}+\frac{\lambda^{*}S^{*}}{\lambda S}\right)+F\left(S,V,L,I,R,P\right), \end{array}$$

where

(58) $$\begin{array}{c} F\left(S,V,L,I,R,P\right)=4-\left(\frac{\lambda^{*}}{\lambda }\frac{S^{*}}{S}\frac{L}{L^{*}}+\frac{L^{*}I}{LI^{*}}+\frac{I^{*}R}{IR^{*}}+\frac{I^{*}P}{IP^{*}}\right) \end{array}$$

balances the right-hand terms of equation (57). Following the approach by [24–26], *F* is a nonpositive function for *S*, *V*, *L*, *I*, *R*, *P* > 0. Thus, *dW*/*dt* < 0 for *S*, *V*, *L*, *I*, *R*, *P* > 0 and is zero if *S* = *S*^∗^, *V* = *V*^∗^, *L* = *L*^∗^, *I* = *I*^∗^, *R* = *R*^∗^, and *P* = *P*^∗^. Therefore, if *R*_*e*_ > 1, model (3) has a unique endemic equilibrium point *E*_1_, which is globally asymptotically stable.

### 3.8. Bifurcation Analysis

Most dynamic systems depend on parameters. Such a dependence implies that any small variation in parameter(s) can have a sudden qualitative change in the behavior of the entire dynamical system. A bifurcation arises when a slight, gradual change in a system's parameter values (the bifurcation parameters) results in a dramatic, qualitative change in the behavior of the system [27]. The local stability attributes of equilibria, periodic orbits, or other invariant sets primarily change at a bifurcation. Several types of bifurcations arise in dynamical systems such as saddle-node, transcritical (forward), pitchfork, and Hopf, to mention a few (for details, see [28]). For this study, we establish the conditions for the presence of either forward or backward bifurcations using the model system (3) developed earlier. In transcritical (forward) bifurcation, two families of fixed points collide and exchange their stability properties. The family that was stable before the bifurcation is unstable after it. The other fixed point goes from being unstable to being stable. The presence of forward bifurcation confirms the eradication of the disease when *R*_0_ < 1. It shows that the DFE is stable when *R*_0_ < 1, and if *R*_0_ crosses unity, then the model admits a unique stable endemic equilibrium. On the other hand, backward bifurcation is a phenomenon that shows the coexistence of stable disease-free and stable endemic equilibrium points when *R*_0_ < 1. In this situation, *R*_0_ < 1 is not a sufficient condition for eliminating the disease. A new critical value (*R*_*c*_ < 1), indicated at the turning point when backward bifurcation occurs, is considered to eradicate the disease. We employ the centre manifold theory presented in [29] to study bifurcation analysis.

**Theorem 5 (see [29]).**

Consider the following general system of ordinary differential equations with a parameter *ψ* : *dx*/*dt* = *f*(*x*, *ψ*), *f* : ℝ^*n*^ × ℝ⟶ℝ and *f* ∈ *ℂ*^2^(ℝ^*n*^ × ℝ), with 0 being an equilibrium point of the system (that is, *f*(0, *ψ*) ≡ 0 for all *ψ*) and assume the following:

A1: *A* = *D*_*x*_*f*(0, 0) = *∂f*_*i*_(0, 0)/*∂x*_*j*_ is the linearization matrix of the system (3) around the equilibrium 0 with *ψ* is evaluated at 0. Simple eigenvalues of *A* include zero, and other eigenvalues of *A* have real components with negative values.

A2: matrix *A* has a right eigenvector *w* and a left eigenvector *v* (each corresponding to the zero eigenvalue).

Let *f*_*k*_ be the *k*th component of *f*

(59) $$\begin{array}{c} \begin{array}{c} a=\Sigma_{k,i,j=1}^{n}v_{k}w_{i}w_{j}\frac{\partial^{2}f_{k}\left(0,0\right)}{\partial x_{i}\partial x_{j}}, \end{array}\\ \begin{array}{c} b=\Sigma_{k,i=1}^{n}v_{k}w_{i}\frac{\partial^{2}f_{k}\left(0,0\right)}{\partial x_{i}\partial \psi }. \end{array} \end{array}$$

The local dynamics of the system around 0 are determined by the signs of *a* and *b*.

- *a* > 0, *b* > 0. When *ψ* < 0 with |*ψ*| ≪ 1, 0 is locally asymptotically stable, and there exists a positive unstable equilibrium; when 0 < *ψ* ≪ 1, 0 is unstable, and there exists a negative, locally asymptotically stable equilibrium
- *a* < 0, *b* < 0. When *ψ* < 0 with |*ψ*| ≪ 1, 0 is unstable; when 0 < *ψ* ≪ 1, 0 is locally asymptotically stable equilibrium, and there exists a positive unstable equilibrium
- *a* > 0, *b* < 0. When *ψ* < 0 with |*ψ*| ≪ 1, 0 is unstable, and there exists a locally asymptotically stable negative equilibrium; when 0 < *ψ* ≪ 1, 0 is stable, and a positive unstable equilibrium appears
- *a* < 0, *b* > 0. When *ψ* changes from negative to positive, 0 changes its stability from stable to unstable. Correspondingly, a negative unstable equilibrium becomes positive and locally asymptotically stable

**Proof**

Suppose *S* = *x*_1_, *V* = *x*_2_, *L* = *x*_3_, *I* = *x*_4_, *R* = *x*_5_, and *P* = *x*_6_; then, the system (3) becomes

(60) $$\begin{array}{c} \begin{array}{c} \frac{dx_{1}}{dt}=f_{1}=\left(1-\rho \right)\Lambda -\left(\mu +\theta +\lambda \right)x_{1},\\ \frac{dx_{2}}{dt}=f_{2}=\rho \Lambda +\theta x_{1}-\mu x_{2},\\ \frac{dx_{3}}{dt}=\lambda x_{1}-\left(\mu +\alpha \right)x_{3},\\ \frac{dx_{4}}{dt}=\alpha x_{3}-\left(\mu +\gamma +\delta \right)x_{4},\\ \frac{dx_{5}}{dt}=\gamma x_{4}-\mu x_{5},\\ \frac{dx_{6}}{dt}=\delta x_{4}-\left(\mu_{p}+\eta -\phi \right)x_{6}, \end{array} \end{array}$$

where

(61) $$\begin{array}{c} \lambda =\beta_{1}x_{4}+\beta_{2}x_{6}. \end{array}$$

Recall that

(62) $$\begin{array}{c} R_{e}=\frac{\alpha \beta_{1}\left(1-\rho \right)\Lambda }{\left(\mu +\alpha \right)\left(\mu +\gamma +\delta \right)\left(\mu +\theta \right)}+\frac{\alpha \delta \beta_{2}\left(1-\rho \right)\Lambda }{\left(\mu +\alpha \right)\left(\mu +\gamma +\delta \right)\left(\mu_{p}+\eta -\phi \right)\left(\mu +\theta \right)}. \end{array}$$

Let *β*_2_ = *kβ*_1_ for *k* ∈ (0, 1) where *k* is a modification factor. Choose *β*_1_ = *ψ*^∗^ as a bifurcation parameter, such that *R*_*e*_ = 1.

(63) $$\begin{array}{c} R_{e}=\frac{\alpha \beta_{1}\left(1-\rho \right)\Lambda }{\left(\mu +\alpha \right)\left(\mu +\gamma +\delta \right)\left(\mu +\theta \right)}+\frac{\alpha \delta \beta_{1}k\left(1-\rho \right)\Lambda }{\left(\mu +\alpha \right)\left(\mu +\gamma +\delta \right)\left(\mu_{p}+\eta -\phi \right)\left(\mu +\theta \right)}=\frac{\alpha \psi^{*}\left(1-\rho \right)\Lambda }{\left(\mu +\alpha \right)\left(\mu +\gamma +\delta \right)\left(\mu +\theta \right)}+\frac{\alpha \delta k\psi^{*}\left(1-\rho \right)\Lambda }{\left(\mu +\alpha \right)\left(\mu +\gamma +\delta \right)\left(\mu_{p}+\eta -\phi \right)\left(\mu +\theta \right)}=1. \end{array}$$

Hence,

(64) $$\begin{array}{c} \psi^{*}=\frac{\left(\mu +\alpha \right)\left(\mu +\gamma +\delta \right)\left(\mu_{p}+\eta -\phi \right)\left(\mu +\theta \right)}{\alpha \left(1-\rho \right)\left(\mu_{p}+\eta -\phi \right)\Lambda +\alpha \delta k\Lambda \left(1-\rho \right)}. \end{array}$$

We linearize the system (60) at (DFE, *ψ*) to get the Jacobian matrix *J* as

(65) $$\begin{array}{c} J\left(E_{0},\psi^{*}\right)=\left[\begin{array}{cccccc} -\mu -\theta & 0 & 0 & -\psi^{*}S_{0}^{*} & 0 & -k\psi^{*}S_{0}^{*}\\ \theta & -\mu & 0 & 0 & 0 & 0\\ 0 & 0 & -\mu -\alpha & \psi^{*}S_{0}^{*} & 0 & k\psi^{*}S_{0}^{*}\\ 0 & 0 & \alpha & -\mu -\gamma -\delta & 0 & 0\\ 0 & 0 & 0 & \gamma & -\mu & 0\\ 0 & 0 & 0 & \delta & 0 & -\mu_{p}-\eta +\phi \end{array}\right]. \end{array}$$

From system (60), it can be shown that the Jacobian matrix (65) has right eigenvalues given by

(66) $$\begin{array}{c} w={\left(w_{1},w_{2},w_{3},w_{4},w_{5},w_{6}\right)}^{T}, \end{array}$$

where

(67) $$\begin{array}{c} \begin{array}{c} w_{1}=-S_{0}^{*}\left(\frac{\left(\mu +\eta -\phi \right)+k\delta }{\left(\mu +\theta \right)\left(\mu_{p}+\eta -\phi \right)}\right)\psi^{*}w_{4},\\ w_{2}=-\theta S_{0}^{*}\left(\frac{\left(\mu +\eta -\phi \right)+k\delta }{\mu \left(\mu +\theta \right)\left(\mu_{p}+\eta -\phi \right)}\right)\psi^{*}w_{4},\\ w_{3}=\frac{\left(\mu +\gamma +\delta \right)}{\alpha }w_{4},\\ w_{5}=\frac{\gamma }{\mu }w_{4},\\ w_{6}=\frac{\delta }{\mu +\eta -\phi }w_{4},\\ w_{4}>0\text{ free variable}. \end{array} \end{array}$$

It can be noted that *w*_3_, *w*_4_, *w*_5_, *w*_6_ > 0 except for *w*_1_, *w*_2_, which are always less than zero.

Also, the left eigenvector *v* = (*v*_1_, *v*_2_, *v*_3_, *v*_4_, *v*_5_, *v*_6_)^*T*^ associated with the zero eigenvalues is obtained as follows:

(68) $$\begin{array}{c} \left(\begin{array}{cccccc} -\mu -\theta & \theta & 0 & 0 & 0 & 0\\ 0 & -\mu & 0 & 0 & 0 & 0\\ 0 & 0 & -\mu -\alpha & \alpha & 0 & 0\\ -\psi^{*}S_{0}^{*} & 0 & \psi^{*}S_{0}^{*} & \mu -\gamma -\delta & \gamma & \delta \\ 0 & 0 & 0 & 0 & -\mu & 0\\ -k\psi^{*}S_{0}^{*} & 0 & k\psi^{*}S_{0}^{*} & 0 & 0 & -\mu_{p}-\eta +\phi \end{array}\right)\left(\begin{array}{c} v_{1}\\ v_{2}\\ v_{3}\\ v_{4}\\ v_{5}\\ v_{6} \end{array}\right)=\left(\begin{array}{c} 0\\ 0\\ 0\\ 0\\ 0\\ 0 \end{array}\right). \end{array}$$

Solving the system (68), we get

(69) $$\begin{array}{c} \begin{array}{c} v_{1}=0,\\ v_{2}=0,\\ v_{3}\;\text{free},\\ v_{4}=\frac{\left(\mu +\alpha \right)}{\alpha }v_{3},\\ v_{5}=0,\\ v_{6}=\frac{k\psi^{*}S_{0}^{*}}{\left(\mu_{p}+\eta -\phi \right)}v_{3}. \end{array} \end{array}$$

Thus, it can be noted that *w*_1_ = *w*_2_ = 0, *v*_3_, *v*_4_, *v*_5_, *v*_6_ > 0.

#### 3.8.1. Computation of Bifurcation Coefficients *a* and *b*

From the normalised model system (60), the associated nonzero partial derivatives of *f* at the disease-free equilibrium is given by

(70) $$\begin{array}{c} \begin{array}{c} \frac{\partial^{2}f_{1}}{\partial x_{1}\partial x_{3}}=0,\\ \frac{\partial^{2}f_{1}}{\partial x_{1}\partial x_{4}}=-\psi^{*},\\ \frac{\partial^{2}f_{1}}{\partial x_{1}\partial x_{6}}=-k\psi^{*},\\ \frac{\partial^{2}f_{3}}{\partial x_{1}\partial x_{3}}=0,\\ \frac{\partial^{2}f_{3}}{\partial x_{1}\partial x_{4}}=\psi^{*},\\ \frac{\partial^{2}f_{3}}{\partial x_{1}\partial x_{6}}=k\psi^{*}. \end{array} \end{array}$$

Computation of *a*:

(71) $$\begin{array}{c} \begin{array}{c} a=\Sigma_{k,i,j=1}^{n}v_{k}w_{i}w_{j}\frac{\partial^{2}f_{k}\left(0,0\right)}{\partial x_{i}\partial x_{j}}, \end{array}\\ a=v_{1}w_{1}w_{3}\frac{\partial^{2}f_{1}}{\partial x_{1}\partial x_{3}}+v_{1}w_{1}w_{4}\frac{\partial^{2}f_{1}}{\partial x_{1}\partial x_{4}}+v_{1}w_{1}w_{6}\frac{\partial^{2}f_{1}}{\partial x_{1}\partial x_{6}}+v_{3}w_{1}w_{3}\frac{\partial^{2}f_{3}}{\partial x_{1}\partial x_{3}}+v_{3}w_{1}w_{4}\frac{\partial^{2}f_{3}}{\partial x_{1}\partial x_{4}}+v_{3}w_{1}w_{6}\frac{\partial^{2}f_{3}}{\partial x_{1}\partial x_{6}},\\ \begin{array}{c} a=\left(v_{3}w_{4}+v_{3}w_{6}k\right)w_{1}. \end{array} \end{array}$$

Since *w*_1_ < 0, then *a* < 0.

Computation of *b*:

(72) $$\begin{array}{c} b=\Sigma_{k,i=1}^{n}v_{k}w_{i}\frac{\partial^{2}f_{k}\left(0,0\right)}{\partial x_{i}\partial \psi^{*}}, \end{array}$$

where

(73) $$\begin{array}{c} \begin{array}{c} \frac{\partial^{2}f_{1}}{\partial x_{1}\partial \psi^{*}}=-\left(x_{4}+kx_{6}\right),\\ \frac{\partial^{2}f_{1}}{\partial x_{4}\partial \psi^{*}}=-x_{1},\\ \frac{\partial^{2}f_{1}}{\partial x_{6}\partial \psi^{*}}=-kx_{1},\\ \frac{\partial^{2}f_{3}}{\partial x_{1}\partial \psi^{*}}=x_{4}+kx_{6},\\ \frac{\partial^{2}f_{3}}{\partial x_{4}\partial \psi^{*}}=x_{1},\\ \frac{\partial^{2}f_{3}}{\partial x_{6}\partial \psi^{*}}=kx_{1}. \end{array} \end{array}$$

Since *v*_1_ = 0, drop all the products associated with the partial derivatives *f*_1_ and obtain

(74) $$\begin{array}{c} b=v_{3}w_{1}\frac{\partial^{2}f_{3}}{\partial x_{1}\partial \psi^{*}}+v_{3}w_{4}\frac{\partial^{2}f_{3}}{\partial x_{4}\partial \psi^{*}}+v_{3}w_{6}\frac{\partial^{2}f_{3}}{\partial x_{6}\partial \psi^{*}}=v_{3}w_{1}\left(x_{4}+kx_{6}\right)+v_{3}w_{4}x_{1}+v_{3}w_{6}kx_{1}, \end{array}$$

at DFE *x*_4_ = *x*_6_ = 0, *x*_1_ = *S*_0_^∗^.

Hence,

(75) $$\begin{array}{c} b=\left(v_{3}w_{4}+v_{3}w_{6}k\right)S_{0}^{*}>0. \end{array}$$

It can be seen that *b* is always positive. Therefore, by Theorem (5) of Castillo-Chavez and Song [29], the local dynamics of the system (60) depends on the sign of the bifurcation constant *a*. Evaluating *a* at bifurcation constant *ψ*^∗^, we get

(76) $$\begin{array}{c} \begin{array}{cc} a= & \frac{\left(\mu +\alpha \right)\left(\mu +\gamma +\delta \right)\left(\mu_{p}+\eta -\phi \right)\left(\mu +\theta \right)\left(v_{3}w_{4}+v_{3}w_{6}k\right)w_{1}}{\alpha \left(1-\rho \right)\left(\mu_{p}+\eta -\phi \right)\Lambda +\alpha \delta k\Lambda \left(1-\rho \right)}<0, \end{array} \end{array}$$

since *w*_1_ < 0. Therefore, with the help of Theorem (5) [29], it can be concluded that since *w*_1_ < 0, a forward bifurcation is guaranteed as *a* < 0 and *b* > 0.

#### 3.8.2. Bifurcation Diagram

The bifurcation diagram shown by Figure 2 represents *I*^∗^ as a function of the basic reproductive number *R*_*e*_.

## 4. Numerical Simulations

In this section, the model system (3) was solved numerically via the Runge-Kutta–fourth-order method and implemented in MATLAB software. Various graphical representations are presented and discussed to validate previously presented analytical findings. Since most parameters were not publicly available, we collected the bulk from the literature and assumed the rest for demonstration purposes. The study used the baseline values of parameters from Table 2 for simulation purposes. Initial values for subpopulations were assumed as follows: *S*(0) = 400, *V*(0) = 300, *E*(0) = 100, *I*(0) = 100, *R*(0) = 100, *P*(0) = 5000.

### 4.1. Effects of Vaccinating Immigrants Only, *ρ*

Here, we discuss how vaccinating immigrants only can help mitigate HA infection. It may be depicted from Figure 3(a) that an increasing vaccination proportion *ρ* decreases the susceptible humans; the same applies for Figure 3(b) where the exposed humans decrease with an increase in vaccination proportion *ρ*. Likewise, in Figure 3(c), infectious humans tend to fall as long as vaccination proportion *ρ* increases, and lastly, in Figure 3(d), the hepatitis A virus population also decreases as a result of the same variation of vaccination coverage *ρ*; this implies that extensive vaccination coverage of the recruits including the newborns is pivotal towards the elimination of HA infection in the community.

### 4.2. Effects of Vaccinating Susceptible Adults Who Missed the First Vaccine, *θ*

It can be observed that some humans who missed the universal compulsory HAV vaccine can receive a vaccine in adulthood at some rate *θ*.  Figure 4(a) shows that an increase in vaccination rate *θ* has an effect of decreasing the susceptible individuals; the same applies to Figure 4(b), where the number of exposed humans fall when the vaccination rate is amplified. Additionally, Figure 4(c) shows that the infectious cases tend to decrease when adult vaccination is maximized, and lastly, in Figure 4(d), the HAV population also falls as a result of the same variety of vaccination parameter *θ*. The results imply that vaccinating adults who missed the first vaccination for some reason seems a critical strategy to control the disease. However, if this effort is not considered, most people may acquire HA infection easily and transmit it to the general population.

### 4.3. Effects of Vaccinating Both Immigrants and Susceptible Adults (*ρ* and *θ*)

It can be observed from Figures 5(a)–5(d) that when one considers vaccinating both immigrants and susceptible adults at the rates *ρ* and *θ*, respectively, there is an abrupt fall in the susceptible, latent, and infectious populations, while hepatitis A virus concentration also remains low. The current results show a dramatic reduction in cases compared to when the same strategies were considered singly. The results indicate that double vaccination offers promising results toward eliminating HA infection in the community.

### 4.4. Effects of Sanitation-Only Strategy

The results from Figures 6(a)–6(c) show that with an improvement in sanitation strategy *η*, there is a substantial decline in HA infection cases. In this strategy, efforts such as water chlorination, boiling drinking water, proper waste disposal, and close personal hygienic practice follow-up may be emphasized with the main agenda of limiting the spread of this disease from the community.

### 4.5. Effects of Combined Vaccination and Sanitation Strategy

In this case, the focus was to assess the role played by combining the two strategies toward eliminating the HA epidemic in the community. From Figures 7(a)–7(d), it can be seen that an increase in vaccination and sanitation strategy has a more significant effect on decreasing the number of HA cases. This has some public health implications when designing initiatives to control the HA epidemic at the national level. One has to consider vaccination and sanitation efforts since this strategy intends to block the primary sources of HA infection, such as contaminated food/water and human-to-human transmission.

### 4.6. Comparison of the Strategies Used to Combat the HAV Epidemic

In this case, a comparison of the strategies used to combat the HAV epidemic is carried out to get a plan that will be most beneficial in controlling the disease. From Figure 8, it can be witnessed that the application of the vaccination-only approach has less effect than the sanitation-only strategy. This implies that vaccinating humans who are less reluctant to adhere to hygienic practices will not be much helpful in mitigating HA infection because even vaccinated humans can acquire the virus when subjected to higher doses of HAV. Vaccination usually reduces the likelihood of getting new infections. On the other hand, sanitation seems to outweigh vaccination; this implies that if sanitation can be implemented perfectly (at higher levels), HA infection elimination is even more possible. Besides, combining the two strategies seems to be the best control strategy. That is to say, to control the HA epidemic in the community, mass vaccination in conjunction with sanitation must be regularly implemented.

## 5. Sensitivity Analysis

We investigate the robustness of model parameters by studying the sensitivity analysis using the effective reproduction number *R*_*e*_. When conducting research, there are usually some errors encountered in data collection methods, so it is vital to consider such deviations. Moreover, the analysis aids in pinpointing which parameters need more attention to manage the disease at an equitable moment. We employ the approach by Chitnis et al. [30] to find a normalized forward sensitivity index. The method uses the reproduction number *R*_*e*_, given by equation (38). One may determine the formula for the normalized forward index such as

(77) $$\begin{array}{c} \Gamma_{\Lambda }^{R_{e}}=\frac{\partial R_{e}}{\partial \Lambda }\times \frac{\Lambda }{R_{e}}=+1,\\ \Gamma_{\rho }^{R_{e}}=\frac{\partial R_{e}}{\partial \rho }\times \frac{\rho }{R_{e}}=-1. \end{array}$$

The remaining set of parameters have the indices as tabulated hereunder.

It can be observed from Table 3 that Γ_*ρ*_^*R*_*e*_^ = −1, which implies that as *ρ* rises, *R*_*e*_ falls. Also, a falling of *ρ* results in a rising of *R*_*e*_, as they are inversely proportional. It can also be witnessed that *θ*, *μ*, *γ*, *δ*, *μ*_*p*_, and *η* are negative; therefore, since they are the reciprocals of *R*_*e*_, which implies that a rise (fall) of any of these particular parameters will cause a fall (rise) in *R*_*e*_.

Conversely, Γ_*Λ*_^*R*_*e*_^ = +1 indicates that increasing *Λ* increases *R*_*e*_ by the same proportion. Similarly, Γ_*Λ*_^*R*_*e*_^ = +1 will drop if *Λ* decreases. In the same manner, *α*, *ϕ*, *β*_1_, or *β*_2_ > 0 are proportional to *R*_*e*_. It means that changing any of these parameters affects *R*_*e*_. One may rearrange the parameters in descending order of their significance from most to least as follows: *Λ*, *ρ*, *θ*, *β*_1_, *δ*, *γ*, *μ*, *μ*_*p*_, *α*, *β*_2_, *ϕ*, and *η*.

## 6. Conclusion

In this work, a nonlinear dynamic mathematical model for the transmission dynamics of HA infection is constructed. Vaccination and sanitation parameters were introduced in the model as control measures. Also, the effective reproduction number was determined via the next-generation matrix technique. The DFE and EE were proven to be locally asymptotically stable when *R*_*e*_ < 1 and unstable otherwise. Also, it was demonstrated that the endemic equilibrium point of the model is globally asymptotic whenever *R*_*e*_ > 1 and unstable otherwise. Bifurcation analysis was established using the centre manifold theory, where it was noted that the model exhibits a forward bifurcation. Epidemiologically, the disease can be eradicated when the reproduction number is kept less than unity. Thus, any efforts, such as vaccination and treatment, affect reproduction negatively, so they could be used to control a disease outbreak.

Besides that, numerical results indicate that applying a single control strategy, like vaccination-only or sanitation-only, may aid in lowering the spread of HA infection. However, it was noted that when both controls were combined, the outcome was even more appealing compared to when each control was considered independently. Thus, there were very few cases when the combined strategy was implemented (see Figure 8).

Additionally, sensitivity analysis was performed to evaluate which parameter(s) play a pivotal role in the transmission of HA infection, such that it could draw serious attention to the mitigation efforts. Parameters catering to a constant recruitment rate *Λ*, vaccination coverage *ρ*, and vaccination rate for susceptible adults *θ* were the most critical parameters to be observed when designing a feasible control strategy. Moreover, human-to-human transmission (*β*_1_) potentially affects disease eruption since it generates higher infections than indirect transmission (*β*_2_). Thus, keeping away from potential sources of HAV will aid in the effective management of the epidemic.

The previous findings have implications for the public and policymakers, especially when designing mitigation strategies; raising vaccination coverage *ρ*, *θ*, and duplication of sanitation efforts *η* will reduce *R*_*e*_ and hence infections. Some initiatives must be set up to ensure that a broad range of people receives compulsory HAV vaccine. Adults who skip vaccination should acquire it because the malady is communicable. Displaced people, the impoverished, and the most disadvantaged groups (women and children, those with disabilities, convicted criminals, refugees, etc.) need fresh drinking water, washroom, and sewage disposal. However, under budgetary constraints, the authorities may opt for single control strategies such as sanitation-only or vaccination-only depending on the extent of the disease in a particular community.

It is worth noting that vaccination and sanitation play important roles in minimizing the possibility of future infections. A vast majority of the literature has documented the success of immunization since ancient times. Thus, there is a need for the world community to support developing countries to alleviate vaccine-preventable diseases by availing vaccines at affordable costs. Also, sanitation infrastructures need to be improved since the model has highlighted its significance in dropping the number of HA cases in the community.

## Figures and Tables

**Figure 1:** A flow diagram for HAV transmission dynamics with some interventions.

**Figure 2:** Forward bifurcation diagram for HAV transmission dynamics model with interventions. When *R*_*e*_ < 1, the disease-free equilibrium is stable. However, when *R*_*e*_ > 1, the disease-free equilibrium is unstable while the endemic equilibrium is stable. The following parameter values were employed for the simulation: *Λ* = 10^3^, *ρ* = 0.5, *θ* = 0.7, *μ* = 0.0130, *α* = 0.0714, *γ* = 0.0476, *δ* = 0.07, *β*_1_ = 0.1, *η* = 0.03, *ϕ* = 0.1, *μ*_*p*_ = 0.9, and *k* = 2.

**Figure 3:** (a–d) show the effects of the vaccination rate *ρ* on different epidemiological classes of HAV transmission dynamics.

**Figure 4:** (a–d) show the effect of HAV vaccination for adults susceptible to different epidemiological classes of HAV transmission dynamics.

**Figure 5:** (a–d) show the effects of vaccination rates *ρ* and *θ* on different epidemiological classes of HAV transmission dynamics.

**Figure 6:** (a–c) Effects of variation of sanitation rate (*η*) on exposed, infectious, and HAV populations.

**Figure 7:** (a–d) show the impacts of the combined vaccination and sanitation strategy on the transmission dynamics of HAV.

**Figure 8:** The comparison of the strategies: sanitation-only, vaccination-only, and a combination of vaccination and sanitation.

**Table 1:** State variables and their definitions for the HAV dynamic model.

Variable	Definition
*S*(*t*)	The number of susceptible humans at a time *t*
*L*(*t*)	The number of latent humans at a time *t*
*I*(*t*)	The number of infectious humans at a time *t*
*R*(*t*)	The number of recovered (immune) humans at a time *t*
*V*(*t*)	The number of vaccinated humans at a time *t*
*P*(*t*)	The number of HA pathogens at a time *t*

**Table 2:** Parameters and their definitions for the HAV dynamic model.

Parameter	Definition	Value	Source
*Λ*	Rate of recruitment of humans into the susceptible class	1000 humans/year	Assumed
*ρ*	A fraction of vaccinated humans	0.7	[11]
*β*_1_	Transmission rate for infectious humans	0.1/year	Assumed
*β*_2_	Effective transmission rate of HAV due to the environment-to-human interaction	0.2/year	Assumed
*δ*	Pathogen shed rate into the water supply or food by infectious humans	80 cells/mL/day	Assumed
*μ*_*p*_	Mortality rate of HA pathogens, including phage degradation	0.83/day	[11]
*η*	Rate at which sanitation measures lead to the death of HA pathogens	2*μ*_*p*_/year	[11]
*γ*	Natural recovery rate for infectious humans (*I*)	1/21/day	[11]
*θ*	Rate at which susceptible humans are vaccinated	0.85/year	[18]
*μ*	Natural human mortality rate	0.00172/year	[18]
*ϕ*	(Maximum) per capita growth rate of HA pathogens	0.73/day	[19]
*α*	Rate at which the latent humans progress to infectious class	1/14/day	[20]

**Table 3:** Parameters and their sensitivity indices.

Parameter	Sensitivity index
*Λ*	+1
*ρ*	-1
*θ*	-0.9818
*μ*	-0.2715
*α*	+0.1538
*γ*	-0.3646
*ϕ*	+0.0174
*δ*	-0.3916
*μ*_*p*_	-0.1565
*β*_1_	+0.8557
*β*_2_	+0.1443
*η*	-0.0052

## Data Availability

The data used to support the findings of this study are included within the article.

## References

[1] Hepatitis A., World Health Organization http://www.who.int/mediacentre/factsheets/fs328/en/.

[2] (1999). Prevention of hepatitis A through active or passive immunization: recommendations of the Advisory Committee on Immunization Practices (ACIP). *MMWR - Recommendations and Reports*.

[3] Stapleton J. T., Lemon S. M. (1994). Infectious Diseases. *(Chapter) Hepatitis A and hepatitis E*.

[4] Trujillo-Ochoa J. L., Viera-Segura O., Fiery N. A. (2019). Challenges in management of hepatitis A virus epidemiological transition in Mexico. *Annals of Hepatology*.

[5] Staes C. J., Schlenker T. L., Risk I. (2000). Sources of infection among persons with acute hepatitis A and no identified risk factors during a sustained community-wide outbreak. *Pediatrics*.

[6] Bianco E., Mariano A., Mele A., Spada E., Tosti M. (2006). Epidemiology of acute viral hepatitis: twenty years of surveillance through SEIEVA in Italy and a review of the literature. *Rapporti Istisan*.

[7] Krugman S., Giles J. P. (1970). Viral hepatitis. *JAMA*.

[8] Koff R. S. (1992). Clinical manifestations and diagnosis of hepatitis A virus infection. *Vaccine*.

[9] WHO (2008). *Hepatitis A*.

[10] Guimaraens M. A. D., Codeço C. T. (2005). Experiments with mathematical models to simulate hepatitis A population dynamics under different levels of endemicity. *Cadernos de Saúde Pública*.

[11] Van Effelterre T. P., Zink T. K., Hoet B. J., Hausdorff W. P., Rosenthal P. (2006). A mathematical model of hepatitis A transmission in the United States indicates value of universal childhood immunization. *Clinical Infectious Diseases*.

[12] Fiore A. E., Wasley A., Bell B. P. (2006). Prevention of hepatitis A through active or passive immunization: recommendations of the Advisory Committee on Immunization Practices (ACIP). *Morbidity and Mortality Weekly Report: Recommendations and Reports*.

[13] Ajelli M., Iannelli M., Manfredi P., degli Atti M. L. C. (2008). Basic mathematical models for the temporal dynamics of HAV in medium-endemicity Italian areas. *Vaccine*.

[14] Ajelli M., Fumanelli L., Manfredi P., Merler S. (2011). Spatiotemporal dynamics of viral hepatitis A in Italy. *Theoretical Population Biology*.

[15] Van Effelterre T., Marano C., Jacobsen K. H. (2016). Modeling the hepatitis A epidemiological transition in Thailand. *Vaccine*.

[16] Brouwer A. F., Zelner J. L., Eisenberg M. C. (2020). The impact of vaccination efforts on the spatiotemporal patterns of the hepatitis A outbreak in Michigan, 2016–18. *Epidemiology*.

[17] Ayouni K., Naffeti B., Ben Aribi W. (2020). Hepatitis A virus infection in Central-West Tunisia: an age structured model of transmission and vaccination impact. *BMC Infectious Diseases*.

[18] Ben Aribi W., Maffei B., Ayouni K. (2022). Global stability and numerical analysis of a compartmental model of the transmission of the hepatitis A virus (HAV): a case study in Tunisia. *International Journal of Applied and Computational Mathematics*.

[19] Edward S., Mureithi E., Shaban N. (2020). *Shigellosis* dynamics: modelling the effects of treatment, sanitation, and education in the presence of carriers. *International Journal of Mathematics and Mathematical Sciences*.

[20] Hethcote H. W., Van Ark J. W. (1987). Epidemiological models for heterogeneous populations: proportionate mixing, parameter estimation, and immunization programs. *Mathematical Biosciences*.

[21] Birkho G., Rota G. C. (1982). Ordinary differential equation. *Stability and Complexity in Model Ecosystems*.

[22] Diekmann O., Heesterbeek J. A. P., Roberts M. G. (2010). The construction of next-generation matrices for compartmental epidemic models. *Journal of the Royal Society Interface*.

[23] Driessche P. V. D., Watmough J. (2008). Further notes on the basic reproduction number. *Mathematical Epidemiology*.

[24] Korobeinikov A., Wake G. C. (2002). Lyapunov functions and global stability for SIR, SIRS, and SIS epidemiological models. *Applied Mathematics Letters*.

[25] Korobeinikov A. (2004). Lyapunov functions and global properties for SEIR and SEIS epidemic models. *Mathematical Medicine And Biology*.

[26] Faye G. (2011). *An Introduction to Bifurcation Theory*.

[27] Korobeinikov A. (2007). Global properties of infectious disease models with non-linear incidence. *Bulletin of Mathematical Biology*.

[28] McCann C. (2013). *Bifurcation Analysis of Non-Linear Differential Equations*.

[29] Castillo-Chavez C., Song B. (2004). Dynamical models of tuberculosis and their applications. *Mathematical Biosciences & Engineering*.

[30] Chitnis N., Hyman J. M., Cushing J. M., Cushing J. M. (2008). Determining important parameters in the spread of malaria through the sensitivity analysis of a mathematical model. *Bulletin of Mathematical Biology*.

